# Application of Nanoparticles in Diagnosis and Treatment of Pancreatic Cancer

**DOI:** 10.1155/2022/7803001

**Published:** 2022-06-06

**Authors:** Juzheng Yuan, Yang Wang, Yang Cao, Shuqiang Yue, Xiao Li

**Affiliations:** ^1^Xi'an Medical University, Xi'an 710021, Shaanxi, China; ^2^Department of Hepatobiliary Surgery, Xijing Hospital, Fourth Military Medical University, Xi'an 710032, Shaanxi, China

## Abstract

**Objective:**

In order to study the application of nanoparticles in the diagnosis and treatment of pancreatic cancer, we retrospectively analyzed pancreatic cancer patients after operation.

**Method:**

60 cases of pancreatic cancer and surgical treatment were selected from our hospital. The time ranged from March 2018 to March 2019. The age ranged from 27 to 81 years. There were 36 males and 24 females, with an average age of 46.23 (7.63) years. Among them, the observation group consisted of nanotube artificial tubes, 16 males and 14 females, while the control group adopted nylon tube, male 18 and female 12. The patient was diagnosed by abdominal CT, and the patient's demographic data and basic clinical data were recorded at the same time.

**Result:**

In this study, 60 patients were divided into groups and compared. The patients underwent surgical resection of pancreaticoduodenum and reconstruction of pancreaticoduodenal papillary duct. Among them, the observation group used nanocomposite artificial tube, while the observation group used nanocomposite artificial tube and placed drainage tube to drain the peritoneal effusion to prevent the effusion from forming in abdominal hypertension and infection. The amount of postoperative bleeding, operation time, and postoperative concomitant symptoms were observed, and the differences between the two materials were analyzed.

**Conclusion:**

The reconstruction of pancreaticoduodenal papillary duct with nanomaterials has certain advantages for postoperative recovery, reduces postoperative complications, reduces the probability of infection, and improves the therapeutic effect.

## 1. Introduction

Nanotechnology is a new technology developed in the 1990s. It is a discussion of the microworld. The microlength of many materials is mostly nano, and many single cells are invisible to the naked eye. The length of 1 nm is equivalent to 10-6 mm. Nanotechnology is to study the application and performance of materials within 100 nm [1]. That is, nanomaterials are accurate to within 10-6 mm to study their properties and applications. So far, China has made some achievements in the application of nanotechnology in other countries. The characteristics of nanotechnology have brought new development directions to many fields such as the application of nanomaterials in medicine, nanochemistry and metrology, and nanobiology [2].

The image of biological cells under the microscope is about 5 microns, and nanomaterials have unique physical and chemical properties, which bring new breakthroughs to the treatment of many diseases in the medical field. Nanomaterials are used more and more in tumor. When materials are made into nanoparticles, their properties also change. The application of nanomaterials in medicine and biology improves the efficiency of diagnosis and treatment [3].

Malignant tumor has become a frequently occurring disease with high mortality. In China, malignant tumor has occurred in all age groups year after year, which has a certain impact on people's life and economy [4]. Although the level of medical science is improving, early diagnosis and intervention can prolong the life cycle of patients. However, the early symptoms of malignant tumors are not obvious so that the patients cannot be diagnosed in time, and the incidence rate of death is high. The age distribution of incidence rate and mortality rate of malignant tumor in China is illustrated in Figure 1.

Incidence rate and mortality rate of malignant tumor are shown in Figure 1, and the incidence rate and mortality rate are 1 : 100000. With the improvement of people's living standards, life expectancy will also be extended, and various diseases will increase accordingly. Malignant tumor has always been one of the diseases endangering people's life safety.

Now people are under great pressure in life; irregular work and rest and unhealthy diet have a certain negative impact on the body, leading to the frequent occurrence of various malignant diseases. Especially for malignant tumors with high mortality, conventional radiotherapy and chemotherapy reduce the human immune system, endanger other organs, and produce great side effects. Targeted therapy with nanomaterials as carriers can inhibit tumor and reduce the adverse effects of drugs. It is the research direction of antitumor therapy after being used in the medical field [5]. When people correctly recognize the existence of tumor, they are not just blindly panic about this disease. How to fight against tumor and obtain more life length and quality of life is the ideological problem of patients and experts in the medical field. Fertility has always been the leading direction of medical research. Increasing the autoimmune system can fight tumor recurrence and metastasis. However, due to the complexity of tumor and human environment, the success rate of the immunotherapy scheme is only 20%. In this paper, nanodrugs can target tumor treatment, deal with the targeted lesions, and improve the immune ability of the local environment so as to improve the overall treatment effect [6].

In particular, the incidence rate of pancreatic cancer is increasing year by year. Its early symptoms are not typical. When obvious symptoms appear, most of them have entered the late stage, with strong invasion, high degree of malignancy, low surgical resection rate, and poor prognosis. It is difficult to diagnose and treat malignant digestive tract diseases. It belongs to one of the malignant tumors with high mortality [7]. Generally, the pancreaticoduodenal papillary duct is reconstructed with a nylon tube after pancreatectomy. In this paper, the nanomaterial is used to replace the nylon tube to reconstruct the pancreaticoduodenal papillary duct, and the nanomaterial is analyzed.

## 2. Data and Methods

### 2.1. Selection of Objects

60 cases of pancreatic cancer and surgical treatment were selected in our hospital from March 2018 to March 2019. The age ranged from 27 to 81 years. There were 36 males and 24 females, with an average age of 46.23 (7.63) years. Among them, the observation group was composed of artificial nanomaterials, 16 males and 14 females, while the control group was treated with nylon tube, male 18 and female 12. All selected subjects need to sign the informed consent form and have the right to know the contents of the study.

### 2.2. Inclusion Criteria

Patients diagnosed with pancreatic cancer confirmed by our hospital were placed in the pancreatic duct for drainage of body fluids. The patient's postoperative physical recovery is ideal, without metastasis and recurrence, normal cardiopulmonary function, free movement and normal language expression ability, clear thinking, civil capacity for their own behavior, and clear expression of their wishes.

Patients who did not place a support tube in the pancreatic duct, had distant organ metastasis, had serious lesions in other organs, had mental disorders and lack of conscious cognition, had incomplete clinical data, refused to cooperate, or were not suitable to participate in the investigation for other reasons were excluded. All patients involved in the investigation had the right to know.

### 2.3. Grouping Method

#### 2.3.1. Control Group

The conventional nylon tube was used to reconstruct the pancreaticoduodenal papillary tube, and the drainage tube was placed to drain the peritoneal effusion so as to prevent the effusion from forming in abdominal hypertension and infection. The amount of postoperative bleeding, operation time, and postoperative concomitant symptoms were observed, and the advantages between the two materials were analyzed.

#### 2.3.2. Observation Group

The pancreaticoduodenal papillary tube was reconstructed with nanocomposite artificial tube, and the drainage tube was placed to drain the peritoneal effusion to prevent the effusion from forming in abdominal hypertension and infection. The amount of postoperative bleeding, operation time, and postoperative concomitant symptoms were observed, and the differences between the two materials were analyzed.

### 2.4. Operation Methods and Observation Indexes

Abdominal exploration was performed through the right upper abdominal incision: tumor details and metastatic cells were found in organs, abdominal diaphragm, stomach, gallbladder, large and small intestines, peritoneum, etc., and gallbladder enlargement occurred. When the stomach colon was cut, it can be seen that the tumor was located in the pancreatic head and often accompanied by lymph nodes. The tumor was separated, the pancreaticoduodenum was removed, and the nanocomposite artificial tube was placed to reconstruct the pancreaticoduodenal papillary tube. At the same time, the drainage tube was placed at the bile intestine and pancreaticointestine to discharge the body fluid and reduce the probability of infection.

After the operation, the patients were replenished with body fluids, supplemented with glucose for nutrition and physical function recovery so as to reduce the possibility of complications, make antibiotics resist the occurrence of infection and other drug intervention, and regularly monitor the physiological indexes of patients to understand the postoperative recovery.

#### 2.4.1. Outcome Measures

Age, sex, preoperative physiological indexes, operation time, total amount of intraoperative bleeding, pancreatic disease, length of hospital stay, abdominal infection, abdominal pressure, other complications, postoperative complications, death, and others.

### 2.5. Statistical Methods

All the observed index data were collected using SPSS22 0 statistical software for statistical analysis, and the measurement data were analyzed with $\bar{x}\pm s$ which indicates that the counting data are expressed in the number of cases and percentage (%), expressed in *χ*^2^ value and *t* value test, and when *T* < 10.000, *P* < 0.05, it means that the data difference is statistically significant, while *T* < 10.000, *P* < 0.01, it means that the data comparison difference is significantly different.

## 3. Results

### 3.1. Comparison of Preoperative Clinical Data between the Two Groups

Before surgery, the clinical data of two groups of patients were compared with age, gender, blood glucose, diabetes, and jaundice. Albumin and total bilirubin were recorded. Then, the general data of these two groups were analyzed by statistical analysis, and the data of Table 1 were obtained.

In Table 1, we can see that there is no statistical significance in the gender and age data of the two groups. In the two groups, the number of patients with hypertension, diabetes, and preoperative jaundice is less. The number of patients with albumin content above 30 g/L is above 90%, while the total bilirubin content in the two groups is below 200 *μ*mol/L. The comparison of all clinical general data between the two groups was not statistically significant (*P* > 0.05).

### 3.2. Comparison of Postoperative Data between the Two Groups

The observation index data of the two groups during and after the operation were retrospectively analyzed, mainly including the amount of bleeding, operation time, length of hospital stay, the proportion of somatostatin used, pancreatic duct diameter, and pancreatic texture, and the data in Table 2 were obtained.

In Table 2, the comparison data of operation time, intraoperative blood loss, and postoperative hospital stay between the two groups can be obtained. The observation index data of patients in the nanocomposite artificial tube group are better than those in the nylon tube group, but the comparison of data on the number of users of somatostatin, pancreatic duct diameter, and pancreatic texture is not statistically significant (*P* > 0.05). After analyzing the data in the above table, we made Figure 2.

In Figure 2, it can be seen clearly that the observation indexes of patients in the observation group are better than those in the reference group. This also shows that the use of nanocomposite artificial tubes in the treatment of pancreatic cancer is beneficial to the recovery of patients and can also help patients discharge faster.

### 3.3. Comparison of Postoperative Complications and Death Data between the Two Groups

Pancreatoduodenectomy is an effective treatment for pancreatic cancer, but any surgical operation has a certain degree of postoperative complications. For this study, the incidence of postoperative complications of pancreatic cancer is very high, and the main complications are biliary fistula, pancreatic fistula, gastric emptying obstruction, gastrointestinal anastomotic leakage, pulmonary complications, and gastrointestinal bleeding. According to the follow-up data and nursing records data of all patients, statistics and analysis are made. The incidence results of postoperative complications in the two groups of patients in Table 3 are obtained.

In Table 3, from the data on the incidence of complications in the two groups, the analysis of the relative ratio of the incidence of complications in the observation group to that in the reference group has a certain statistical significance, and although both groups of patients have a certain degree of complications, they will not cause deaths.  Figure 3 is made according to the complication data of the two groups of patients.

In Figure 3, the incidence of complications in patients with nanocomposites is lower than that in patients with nylon tubes, which shows that the use of nanocomposites can effectively reduce the incidence of complications and reduce the postoperative pain of patients.

### 3.4. Comparison of Postoperative Pancreatic Fistula Data between the Two Groups

Pancreatic fistula is one of the most serious complications of pancreatic duct resection for pancreatic cancer surgery because pancreatic fistula after the operation can cause pancreatin to activate in vivo, and the activated pancreatin is highly corrosive, which will corrode the anastomotic stoma of the patient, resulting in further corrosion of pancreatic enzymes into the abdominal cavity, resulting in bleeding and infection. The data in Table 4 are the incidence of pancreatic fistula in two groups of patients.

In Table 4, it can be seen that the severity of pancreatic fistula in patients is divided into three levels, of which grade A is the lightest and grade C is the most serious. It can be seen from the data in the table that the overall incidence of pancreatic fistula in the nanocomposite artificial tube group is lower than that in the nylon tube group, and for each grade, the number of patients in the nylon tube group is much higher than that in the observation group.  Figure 4 is made according to the incidence data of pancreatic fistula in the two groups.

In Figure 4, it can be seen that the comparison of the incidence of pancreatic fistula complications between the two groups is statistically significant, and the incidence of pancreatic fistula in the observation group with nanocomposites is much lower than that in the reference group, which shows that the artificial tube made of nanocomposites instead of nylon tube can effectively reduce the incidence of postoperative pancreatic fistula.

## 4. Discussion

Pancreatic cancer is a malignant tumor of the digestive tract. Its early symptoms are not obvious. Some people may suffer from abdominal pain, abdominal distention, nausea, and vomiting. It often causes swelling of organs and gallbladder. Some people will have jaundice. Conventional blood and urine can not be diagnosed. When they are found, they often suffer from other organ metastases, resulting in delayed condition and subsequent treatment.

Conventional tumors are usually treated by surgical resection and radiotherapy and chemotherapy, but radiotherapy and chemotherapy do great harm to the human body and have obvious side effects. According to relevant data, the survival period of pancreatic cancer patients without surgical treatment is relatively short, and even if the survival rate of five years after the operation is only about 5%, it is a malignant tumor with higher mortality.

The emergence of polymer materials provides a new research direction for medical research. The application of nanomaterials brings hope to cancer treatment. At present, although it is impossible to cure malignant tumors for the time being, there is still room for development in improving the treatment effect and reducing the negative impact. The early diagnosis of some tumor diseases with high malignancy is extremely important. Early intervention of the lesions is helpful to the recovery of the disease. The use of nanomaterials as magnetic resonance contrast agents in the diagnosis of pancreatic cancer provides a new direction for the early diagnosis of pancreatic cancer [8].

The early diagnosis and intervention of malignant tumors play a great role in the disease and contribute to the improvement of the disease and the survival rate. Molecular imaging can detect the abnormal phenomenon of cell level in the early onset of the disease and diagnose some recessive diseases as soon as possible. The application of nanomolecular imaging technology in the early diagnosis of pancreatic cancer provides the basis for the early diagnosis of pancreatic cancer [9].

Pancreatic cancer is a malignant tumor with poor prognosis. Although huge investment has been made in the early diagnosis and comprehensive treatment of pancreatic cancer, the survival rate of tumor patients has not been significantly improved. With the synthesis and application of multifunctional nanoparticles, nanotechnology will quickly become one of the most promising methods for the diagnosis and treatment of pancreatic cancer. The application of nanomaterials brings not only new challenges and opportunities to the medical field but also good news to patients [10]. The early concealment of pancreatic malignant tumor brings some difficulties to the diagnosis so that its mortality remains high [11]. Early diagnosis and intervention can improve the prognosis after the operation. Nanomaterials bring new research directions to the early diagnosis of pancreatic malignant tumor, and the application of nanomaterials during operation brings a safe and effective way to cancer treatment and provides a basis for medical development.

## 5. Conclusion

Scientific and technological progress has driven many polymer materials to be recognized and applied to various fields. The application of nanomaterials has brought many exploitable prospects to the medical field, especially in medical imaging and early diagnosis, which provides a basis for the diagnosis of some highly hidden malignant tumors [12]. Advances in the field of medicine have made malignant tumors no longer exist like death, endangering human life and making patients miserable [13]. The study found that the reconstruction of pancreaticoduodenal papillary duct with nanomaterials has certain advantages for the postoperative recovery of patients, reduces postoperative complications, reduces the probability of infection, and improves the treatment effect. Although the five-year survival rate of patients with pancreatic cancer is relatively low, improving the quality of life and prolonging the life cycle of patients are the current treatment objectives of pancreatic cancer to reduce the physiological pain of patients. It is believed that with the development of science and technology, the higher the cognition of new materials, there will be more and more applications of nanoparticles in clinical medical research.

## Figures and Tables

**Figure 1:** Age distribution of incidence rate and mortality rate of malignant tumor in China.

**Figure 2:** Comparison of postoperative clinical data and results between the two groups.

**Figure 3:** Comparison of complication rates between the two groups.

**Figure 4:** Comparison of the incidence of pancreatic fistula between the two groups.

**Table 1:** Comparison of general data and results before operation between the two groups.

Index classification		Nanocomposite artificial tube group	Nylon tube group	*t* value	*P* value
Age	≥60	11 (36.67%)	13 (43.33%)	7.654	0.348
	＜60	19 (63.33%)	17 (56.67%)	6.325	0.631

Gender	Male	16 (53.335)	18 (60%)	4.367	0.534
	Female	14 (46.67%)	12 (40%)	7.148	0.324

Hypertension		10 (33.33%)	11 (36.67%)	6.358	0.897
Diabetes		6 (20%)	8 (26.675)	5.541	0.547
Preoperative jaundice		5 (16.67%)	6 (20%)	5.327	0.657

Preoperative albumin (g/L)	≥30	27 (90%)	29 (96.67%)	7.364	0.357
	＜30	3 (10%)	1 (3.33%)	6.396	0.571

Total bilirubin (*μ*mol/L)	≥200	3 (10%)	5 (16.67%)	6.365	0.368
	＜200	27 (90%)	25 (83.33%)	7.219	0.589

**Table 2:** Comparison of postoperative clinical data and results between the two groups.

Index classification		Nanocomposite artificial tube group	Nylon tube group	*t* value	*P* value
Operation time (h)		5.24 ± 1.64	6.84 ± 1.53	3.654	0.032
Intraoperative bleeding volume (ml)		164.94 ± 53.97	197.84 ± 65.38	3.321	0.038
Postoperative hospital stay (d)		20.65 ± 10.64	26.54 ± 11.61	3.847	0.029
Somatostatin		79.36%	75.58%	6.954	0.364

Pancreatic duct diameter (mm)	≥3	65.34%	58.95%	6.323	0.548
	＜3	34.66%	41.05%	6.414	0.267

Pancreatic texture	Soft	53.64%	60.36%	7.036	0.367
	Hard	46.36%	39.64%	7.214	0.585

**Table 3:** Comparison of postoperative complications between the two groups.

Classification of complications	Nanocomposite artificial tube group	Nylon tube group	*t* value	*P* value
Biliary fistula	3 (10%)	7 (23.33%)	5.647	0.035
Gastrointestinal anastomotic fistula	1 (3.33%)	5 (16.67%)	5.149	0.025
Gastric emptying disorder	2 (6.67%)	9 (30%)	5.367	0.026
Pulmonary complications	4 (13.33%)	14 (46.67%)	5.021	0.042
Gastrointestinal bleeding	2 (6.67%)	8 (26.67%)	5.034	0.033
Reoperation	1 (3.33%)	5 (16.675)	5.514	0.031
Death	0 (%)	0 (%)	5.241	0.026

**Table 4:** Comparison of the incidence of pancreatic fistula between the two groups.

Grouping	Level A	Level B	Level C
Nanocomposite artificial tube group	2 (6.67%)	2 (6.67%)	1 (3.33%)

Nylon tube group	5 (16.675)	6 (20.00%)	9 (30.00%)

*t* value	7.658	6.523	7.854

*P* value	0.034	0.025	0.021

## Data Availability

The data underlying the results presented in the study are available within the manuscript.
